This article has been retracted.

# Computer-Assisted Quantitative Analysis of Skeletal Muscles of Snowboarding Parallel Giant Slalom Athletes after Exercise Based on Artificial Intelligence and Complex Networks

**DOI:** 10.1155/2022/9755658

**Published:** 2022-04-22

**Authors:** Haiqiang Yu, Fei Yang, Jin Wang

**Affiliations:** ^1^School of Physical Education, Liaoning Normal University, Dalian, 116029 Liaoning, China; ^2^Department of Physical Education and Research, Dalian Medical University, Dalian, 116044 Liaoning, China

## Abstract

The snowboarding project has the characteristics of high risk and high technical level. The current publicity level is not high, and the number of participants is also very limited. Another potential advantage medal breakthrough project that is expected to be achieved in the Winter Olympics has received a lot of attention, creating favorable opportunities for the promotion and development of this project in China. The event requires good special physical support, skeletal muscle contraction is the body to produce motor function, and special physical training and recovery are key factors for athletes to obtain excellent results in the competition. This article is aimed at performing ultrasonic quantitative analysis on the skeletal muscles of skiers after exercise based on artificial intelligence and complex networks and at studying the skeletal muscle conditions of snowboarders after exercise, so as to provide a certain theoretical basis for coaches in future scientific training. Based on a large amount of literature, this paper uses variational optical flow calculation and split Bregman method to solve the typical HS model, L1-L2 model, and L1-high-order model, respectively, and uses the motion estimation method to describe the movement of muscles. An experiment was designed to collect ultrasound images of the gastrocnemius and quadriceps muscles during contraction. In addition, a motion target positioning algorithm was used to obtain some motion parameters, which provided direct help for athletes in rationally arranging training load and scientific training. The experimental results in this paper show that the muscle motion features extracted from the ultrasound sequence images can quantitatively express a lot of important information about the skeletal muscle motion form and function and have potential practical application value. And the different invariants of each type of ski trajectory vary greatly, floating between 1.5429 and 7.6759.

## 1. Introduction

### 1.1. Background

Skeletal muscle is generally fixed by tendons at both ends of the bone and is an important tissue that constitutes the human body. The human body has about 600 skeletal muscles, which control basic human activities including flexion, extension, and extension. Skeletal muscle contraction is the driving force for the human body to produce sports functions, and its strength and endurance directly affect human body performance during exercise. In order to understand the mechanics of human movement, it is particularly important to study the structure, function, and movement characteristics of human muscles. Because the composition of muscles is very complex and the exercise process is complex and diverse, quantitative analysis and multilevel analysis of the functional state of muscles are the focus and difficulty of current research. This includes understanding how muscles control the degree of strength, whether all muscle fibers have the same function, and how to obtain as much information as possible from a single muscle of the human body at the same time and perform comprehensive processing. These are all issues worthy of attention. In addition, the snowboard parallel giant slalom is an emerging winter sports project in China in recent years. It has been developed for less than 7 years. It can be said that the coaches of this project are in the development and learning stage. They need to have more special physical training and the regular characteristics of the project development.

In in-depth understanding, the snowboard parallel giant slalom is a relatively high-tech sports event, which is very ornamental, exciting, and very thrilling. The snowboard parallel giant slalom track is very long, the flag gate is set far, and the downhill speed is fast. Two athletes start at the same time, which requires higher athletes' muscle strength and speed quality.

### 1.2. Significance

At present, Chinese snowboard parallel giant slalom skiing is in the initial development stage of the project, and the research process in many fields is still very slow, and some areas are even blank. Through consulting and researching a large amount of literature, coaches and scientific researchers have conducted some research and practice in determining the content of land special training, the selection of training methods, and the application of training methods, and certain progress has been made. It was found that there are not many related articles about the monitoring and evaluation of the effects of athletes' land training through biomechanical means. There are no articles about the monitoring and evaluation of the effects of snowboarding parallel giant slalom athletes on water and land training through biomechanical means. According to the experimental results, the athlete's flexor and extensor strength can be seen. If a certain part of the muscle strength is found to be weak, strengthen the exercise in time to reduce sports injuries. This set of evaluation methods can also objectively evaluate the feasibility of land training plans and programs from the perspective of biodynamics, so as to provide a bit of reference for the selection of the best training program for snowboard parallel giant slalom trainers. This research lays the foundation for follow-up in-depth and comprehensive research and provides a certain reference for innovative research on related topics.

### 1.3. Related Work

The physical training of the snowboard parallel giant slalom has played an important role in ensuring the athlete's physical fitness during training and competition and has played a positive role in promoting technical learning. General physical training is the foundation, and special physical training is the key. Minniti et al. proposed that central nervous system diseases and musculoskeletal diseases often involve skeletal muscles. They used real-time shear wave elastography (SWE) to accurately and quickly quantitatively evaluate the strength and stiffness of individual muscles; it uses the probe to emit safe acoustic radiation pulses, which are continuously focused on different depths of the tissue to cause tissue particles to vibrate and generate transverse shear waves, allowing for accurate quantitative measurement of the shear waves in the tissue being examined, thus achieving real-time accurate monitoring of the shear wave propagation process within the swept section, and concluded that SWE assists in skeletal muscle diseases. The diagnosis has a greater role [1]. Jang et al. compared the metabolic patterns before and after exercise. By using orthogonal partial least squares discriminant analysis (OPLS-DA) and variable importance maps for multivariate data scoring based on metabolic profiles, for orthogonal partial least squares discriminant analysis, a linear regression model and least squares are used to project continuous variables orthogonally (orthogonal) to the latent structure, thus separating the variables into those that are predictable and those that are irrelevant, with the first latent variable explaining the common variation between *X* and *Y* and the second followed by latent variable is irrelevant (orthogonal) to *Y* in *X* variation. In case of discontinuous variables, it is possible to classify the different classes. We found that the patterns of metabolites in the athletes' muscles, plasma, and urine have changed before and after exercise. However, specific content relationships have not been derived, so they have not been adopted on a large scale [2]. Ju et al. proposed that mitochondrial homeostasis is strictly regulated by two main processes: mitochondrial biogenesis and mitochondrial degradation caused by autophagy (mitophagy). The authors measured autophagy flux and showed that autophagy plays an important role in mitochondrial biogenesis. This coordination between these opposing processes is involved in the adaptation of cells to endurance exercise training [3]. Czell et al. pointed out that ultrasound has become a reliable method for detecting fasciculation. By taking 50 samples and using ultrasound for 120 seconds, 45 minutes, 50 samples of 3 arm and 3 leg muscles were investigated, and the conclusion was healthy. The muscles above the knees of the subject may experience fasciculation [4]. Goldfain et al. proposed that the combination of phase contrast imaging technology and tomographic reconstruction can quickly measure the ultrasonic field propagating in the water. This technology shows that phase contrast imaging can accurately measure the ultrasonic field with a frequency of up to 20 MHz and a pressure amplitude close to 10 kPa and optical imaging. The extension of measurement to high ultrasound frequencies can promote the quantitative application of ultrasound measurement in nondestructive testing and medical treatment and diagnosis (such as photoacoustic imaging) [5]. Korf et al. proposed that the expression of genes responsible for the synthesis of essential proteins regulates calcium ion balance and ultrastructural characteristics of fast muscles (m. extensor digitorum (EDL)) and slow muscles (m. soleus (SOL)) in skeletal muscles under long-term exercise. The expression will change. Through the establishment of experimental models and the use of electron microscopes, it is shown that the adaptation of SOL muscle is related to the structural rearrangement of the mitochondrial apparatus, while the adaptation of EDL muscle is the removal of calcium from the sarcoplasm by Ca-ATPase and the retention of calcium by calsequestrin caused in the sarcoplasmic reticulum [6]. Although the analysis is in place, there are some problems in the analysis process that requires attention.

### 1.4. Innovation

The innovation of this article is as follows: (1) The first one is the innovation of the topic selection angle. This article is a new perspective from the perspective of topic selection. At present, there are not many researches that integrate artificial intelligence, computer assistance, snowboarding, physical fitness, and skeletal muscle. It is of exploratory significance. (2) The second one is the innovation of research methods. This paper proposes variational optical flow calculation, split Bregman method, moving target positioning algorithm, etc., which have high theoretical value and exploratory significance. (3) The other one is the innovation of project practice. The results of the project have created a favorable opportunity for the promotion and development of the project in China and at the same time provide part of the theoretical basis for the training of athletes in the future.

## 2. Motion Estimation Algorithm

### 2.1. Variational Optical Flow Calculation

The optical flow method makes an important method for motion image sequence analysis, where accurate estimation is required in many motion analysis applications, and the variational-based optical flow calculation can meet this requirement. We use function *f* : *ϖ* × *P*⟶*Μ* to represent the image sequence, where *ϖ*⊆*P*^2^ represents the image domain [7], which is rectangular in most cases, and *M*⊆*P* represents the time domain. The problem to be solved is to calculate the motion field of two image frames *D* and *D* + 1 at two adjacent moments. The two components of this motion field are represented by *s*, *a* : *ϖ*⟶*P*.

The variational optical flow calculation based on the energy function can be expressed as the following form:

(1) $$\begin{array}{c} \underset{s,n}{\min}\;E\left(s,n\right)=\int \int_{\varpi }\underset{\text{Data}}{\underbrace{D\left(\partial^{k}f,s,n\right)}}+\underset{\text{Smoothness}}{\underbrace{\lambda a\left(\nabla f,\nabla u,\nabla v\right)dxdy}}. \end{array}$$

Below, we derive data items for different characteristics based on different assumptions. The first natural idea is to keep the gray value constant; that is, there is

(2) $$\begin{array}{c} d\left(x,y,t\right)=d\left(x+u\left(x,y\right),y+v\left(x,y\right),t+1\right). \end{array}$$

So we assume that the spatial derivative of *d* can also remain unchanged, and we get

(3) $$\begin{array}{c} \nabla d\left(x,y,t\right)=\nabla d\left(x+u\left(x,y\right),y+v\left(x,y\right),t+1\right). \end{array}$$

In order to limit the problem to the convex function domain [4], we carry out a first-order Taylor expansion of *d* and ∇*f* at time *D*. First, combine their sum of squares to construct a data item:

(4) $$\begin{array}{c} Q_{\text{Data}}^{1}\left(u,v\right)={\left(f_{x}c+f_{y}h+\text{ft}\right)}^{2}+\gamma {\left(f_{xx}c+f_{xy}h+f_{xt}\right)}^{2}, \end{array}$$

where *λ* > 0 represents the weight between the two hypotheses [8]. The above formula is convex and smooth, so it has good properties, but it is not good for edge processing. Similarly, construct data items:

(5) $$\begin{array}{c} Q_{\text{Data}}^{2}\left(u,v\right)=\left\|f_{x}c+f_{y}h+\text{ft}\right\|+\gamma \left(f_{xx}c+f_{xy}h+f_{xt}\right). \end{array}$$

*Q*_Data_^2^ is more stable than *Q*_Data_^1^, but its disadvantage is that its absolute value is not differentiable at 0 point.

### 2.2. Split Bregman Method

When solving an optimization problem containing *W*_1_, the Bregman method has the advantages of high efficiency, constant regularization parameter *λ*, and stability of the algorithm [9]. However, in Bregman iteration, each iteration needs to solve a complex variational problem, which increases the numerical difficulty. At the same time, we should also see that the standard Bregman method deals with constrained optimization problems, while the optimization problem to be dealt with in this article is unconstrained. This makes us choose a split algorithm of the standard Bregman method: split Bregman method (split Bregman Method), which was proposed by Goldstein and Osher when dealing with image restoration problems in 2009. First, consider the following optimization problem with *W*_1_ terms:

(6) $$\begin{array}{c} \underset{v}{\min}\;F\left(v\right)+{\left|Xv+b\right|}_{1}. \end{array}$$

The idea of splitting the Bregman method is mainly to introduce an additional variable to separate the differentiable and nondifferentiable terms in the model and then to minimize them separately [10]. If so, the problem can be transformed into the following constrained optimization problem:

(7) $$\begin{array}{c} \underset{s,d}{\varpi }H\left(v\right)+{\left|d\right|}_{1}s.t.d=\beta u. \end{array}$$

By introducing parameters *ε*, the above problem can be transformed into the following unconstrained optimization problem:

(8) $$\begin{array}{c} \underset{s,v}{\min}\;H\left(v\right)+{\left|d\right|}_{1}+\frac{\mu }{2}{\left\|d-\alpha u-n^{k}\right\|}_{2}^{2}. \end{array}$$

Using the idea of compact Bregman iteration, the following iterative method can be used to solve the above optimization problem:

(9) $$\begin{array}{c} \left\{\begin{array}{c} \left(v^{k+1},h^{k+1}\right)=\arg\min H\left(u\right)+{\left|d\right|}_{1}+\frac{\partial }{2}{\left\|d-\beta u-b^{k}\right\|}_{2}^{2},\\ n^{k+1}=n^{k}+b+\eta b^{k+1}-f^{k+1}. \end{array}\right. \end{array}$$

The first formula in the above formula is convex with respect to *v* and *n*, so the problem can be divided into the following subproblems:

(10) $$\begin{array}{c} \left\{\begin{array}{c} f^{kj+1}=\underset{v}{\arg\min H\left(v\right)+\frac{\alpha }{2}{\left\|f^{kj}-\alpha v-b^{k}\right\|}_{2}^{2}},\\ f^{kj+1}=\underset{k}{\arg\min{\left|d\right|}_{1}+\frac{\mu }{2}{\left\|d-\alpha u^{kj+1}-b^{k}\right\|}_{2}^{2}},\\ n^{k+1}=n^{k}+b+\eta b^{k+1}-f^{k+1}. \end{array}\right. \end{array}$$

For *y* ∈ *β* and *∂* > 0, threshold operators [11] are defined as follows:

(11) $$\begin{array}{c} \text{shrink}\left(y,\alpha \right)=\mathrm{sgn}\left(y\right)•\max\left(\left|y\right|-\partial ,0\right). \end{array}$$

For function *f* : *Q*^*n*^⟶*Q*, it has the following form:

(12) $$\begin{array}{c} f\left(x\right)={\left|x\right|}_{1}+\frac{\alpha }{2}{\left\|x-b\right\|}_{2}^{2} \end{array}$$

When solving optimization problems containing *W*_1_ nondifferentiable term, the threshold operator has been widely used in many fields of image processing due to its simple programming, small memory occupation, and relatively easy implementation. It needs to be pointed out that when dealing with similar optimization problems containing *W*_1_ items; the following conclusions are made:

(13) $$\begin{array}{c} \underset{v}{\min}\;H\left(v\right)+{\left\|\alpha v+b\right\|}_{2}. \end{array}$$

Among them, *∂* > 0, *b* ∈ *R*, and the condition for the function *f* to obtain the minimum value is *x* = *g*shrink(*b*, (1/*β*)), where

(14) $$\begin{array}{c} g\text{shrink}\left(b,\lambda \right)=\max\left({\left\|c\right\|}_{2}-\lambda ,0\right)\frac{\beta }{{\left\|b\right\|}_{2}}. \end{array}$$

### 2.3. Moving Target Positioning Algorithm

When there are multiple observation stations measuring the target angle, the position of the target can be estimated using the least squares positioning algorithm. The Least Square Estimator (LSE) is a parameter estimation result given from the perspective of data fitting. It gives parameter estimates that conform to the “best fit” [12, 13] based on the existing observation data and models. From a mathematical point of view, it can also be regarded as an approximate solution to an overdetermined system of equations. Usually, we define the sum of squares of the error between the observed value and the model estimate as the minimization criterion.

(15) $$\begin{array}{c} R_{\text{LSE}}=\underset{\lambda }{\arg\min}J\left(\lambda \right), \end{array}$$

in

(16) $$\begin{array}{c} J\left(\lambda \right)={\left[m-f\left(\pi \right)\right]}^{\eta }\left[m-f\left(\beta \right)\right]. \end{array}$$

Function 1 represents the numerical relationship between the measurement model and the unknown parameters. If the functional relationship can be written as linear form 2, then the formula (16) is sorted into

(17) $$\begin{array}{c} F\left(\lambda \right)=m^{T}m-2m^{\alpha }H\gamma +\partial^{\gamma }H^{\eta }H\gamma . \end{array}$$

Let its first-order differential equation be zero to find the least squares estimator:

(18) $$\begin{array}{c} \lambda_{\text{LSE}}={\left(G^{T}WH\right)}^{-1}H^{T}m. \end{array}$$

It is worth noting that the premise of the above formula is that the matrix *H*^*T*^*m* in the brackets is invertible [14]. And only when all observations are Gaussian variables with independent and identically distributed (independent and identically distributed), *λ*_LSE_ is the effective best linear unbiased estimator [15] (Best Linear Unbiased Estimator (BLUE)).

Further, if the components of the observation are independent of each other but have different variances, add a weighting matrix *Q* = *E*_*m*_^−1^ to modify, such as

(19) $$\begin{array}{c} J\left(\lambda \right)={\left[m-f\left(\lambda \right)\right]}^{T}W\left[m-f\left(\kappa \right)\right]. \end{array}$$

Then, in the minimization criterion, we determine its contribution to the fitting according to the variance of the observations [16]. Similarly, for linear model *f*(*γ*) = *Hλ*, the weighted least squares estimator of unknown vector *λ*° also satisfies

(20) $$\begin{array}{c} \lambda_{\text{WLS}}={\left(H^{T}WH\right)}^{-1}H^{T}Wm. \end{array}$$

This also shows that it is of practical significance to use the sum of squares of errors as the criterion of least squares estimation [17, 18].

## 3. Establishment of MRF Model

### 3.1. Collection and Processing of Experimental Data

The processing and flow of data is an important part of the system. The following uses a data flow chart to briefly show the flow and processing of data in the system [19–22]. The data flow chart is divided into the top chart, the 0-level chart [23], and the 1-level chart. Figures 1 and 2 are displayed in layers from the top level to the first level and from the outside to the inside. Among them, there are 6 subgraphs in the level 1 chart. From Figure 1 to Figure 2, the search center of 1 query is decomposed from the level 0 chart, as shown in Figures 1 and 2.

The data flow diagram-0 level diagram divides the center of a problem into the following six subparagraphs: in the health and medical center sports, the database and the physical state data of the relevant players are searched in different locations [2] and the sports competition data processing center [24]. In games such as recovery speed and acceleration, the players' various points are in the database and pass the list. In addition, according to the requirements of users, it is possible to intercept the data of a specific time period or Gyeongju unit and run the speed statistics space within a specific time. By registering the player's position and direction through the bass, it is also possible to restore the player's trajectory and speed data at different times during the game. The player video management center can be called and recorded through the camera [25], and the camera can be played according to the requirements of users and managers. The processing center environmental data searches the database for environmental data (snow field temperature, snow surface humidity, wind speed, etc.) and provides feedback to users at any time according to statistical charts of data changes. The data processing center can add, delete, and modify data according to the requirements of operators and users. Players can only see part of their data and information for modification. The coach can modify his information based on the driver's data. The administrator must have the highest authority to perform all functions.

### 3.2. MRF Model for Reliability Analysis of Motion Vector

In the searched motion vector field, the motion vector information of each block [1] is characteristic data, and its reliability classification can be regarded as a random variable, and the value of the variable is the reliability category of the motion vector. Reliability is divided into three categories here: reliable, wrong matching, and multiple matching, where 0 represents the reliable category, 1 represents the wrong matching category, and 2 represents the multiple matching category. The entire motion vector field can be regarded as a Markov random field. It is believed that the reliability of each motion vector is only related to the reliability of its neighboring motion vectors and has nothing to do with the reliability of other motion vectors.

Potential energy function *T*_2_(*f*_*i*_, *f*_*r*_) describes the constraint relationship between two adjacent motion vectors. From the previous analysis, it can be seen that this constraint relationship is not only related to the adjacent position of the two motion vectors but also related to the difference of the motion vector itself, so it cannot directly adopt the traditional ISING model or Potts model [26]. That is to say, for different values of *i* and *r*, the coupling coefficient *β* is different, and for fixed values of *i* and *r*, the coupling coefficient *β* is also related to the difference distribution of the specific motion vectors of *i* and *r*, that is, with *i* and *r* The specific value of is related to the probability when different motion vectors are different. When there is a certain difference, the greater the probability of the specific values of *i* and *r*, the stronger the mutual constraint, and vice versa.

For this reason, the probability statistics of the specific values of adjacent *i* and *r* when different motion vectors are different are made here. The experiment performed statistics on 138 image pairs in the database, and the difference between the two motion vectors is represented by their modulus. The three cases are, respectively, counted. The first case is that the adjacent point elements *i* and *r* are both reliable. The second case is that the adjacent point elements *i* and *r* are multiple matches. In fact, there is the last case that one of the adjacent point elements *i* and *r* is mismatched. Considering the mismatched SVM classification is correct, the rate is high enough, and adjacent mismatches do not have Markov properties, so they are not considered here.

Among them, the abscissa indicates the ordering size of the difference, and the ordinate indicates the probability distribution of the reliability markers at this time. The statistical results of the two cases are shown in Figures 3 and 4.

For the convenience of calculation, the probability distributions of the above reliability markers are merged in sections, and if the probability of similar motion vector differences is small, they are merged into the same probability. It can be seen from the figure that when the difference between two adjacent motion vectors is the smallest, that is, (1, 1), the probability that the two point elements are both reliable classes is about 0.8, and there is a probability of 0.06 for both of them. It belongs to the multimatching category, and the probability that the reliability of two points are not the same is almost zero. Once again, when the difference between two adjacent motion vectors is small, their reliability is very likely to be consistent. And when two adjacent motion vectors are very different, the probability that they are both reliable classes is almost zero. In fact, most of the cases at this time are in the situation where the two motion vectors are mismatched or multimatched. This is also the previous analysis of the spatial relationship of the motion vector verified.

### 3.3. Torso Isometric Muscle Strength Test

#### 3.3.1. Test Instrument

TORSOLINE is a series of body diagnosis and training institutions produced by German ERGO-FIT Company. Because of simple, fast, accurate, and effective diagnosis and accurate and easy-to-control training, it is widely used at present. TORSOCHECK is a diagnostic mechanism used in the TORSOLINE combination, which has the function of testing and analyzing the muscles displayed in all directions of the spine. It includes six movements, namely: flexion and extension in the sagittal plane, flexion to the left and right in the coronal plane, and rotation to the left and right in the horizontal plane. The test results of TORSO CHECK reflect the defect and imbalance of muscle strength.

#### 3.3.2. Test Methods

The tester opens the computer supporting the instrument, connects the required sensors, opens the program, enters the required information, and enters the test interface. As the subjects completed their actions, an ultrasound instrument equipped with a 12 MHz linear array probe was used to obtain ultrasound images of the gastrocnemius muscle. The ultrasound probe is placed on the gastrocnemius muscle belly and parallel to its longitudinal direction. The ultrasound couplant is used in the middle to closely fit the ultrasound probe. The ultrasound probe is fixed on the calf through the self-made multiangle bracket, and the position is adjusted to make it. Muscle fibers are clearly seen in the ultrasound image, as shown in Figure 5.

Let the subject sit on the “TORSO CHECK,” and while contacting the lumbar spine and backrest, fix the subject in four directions: front, back, left, and right, and fix the upper position of the shoulder sensor 5 cm below the acromion

When the subject is sitting still, pull the right hand with the left hand and the left hand with the right hand

The tester issued a password to make the subject apply the maximum isometric contraction force in 8 directions, including front, back, left, right, left, and right, for 10 seconds each time, 4 times in total. So subjects are familiar with the feeling of exertion

In accordance with the computer program and operating specifications, complete 4 times of maximum isometric contraction strength test of 15 seconds each time. There should be an interval of 1 minute between each test and the last test. During each test, the test personnel use the following: “Come on! Hard! Very good! Hold on!” Encourage the subject with words

Complete the test, release the fixation, relax the subject, and save the data

#### 3.3.3. Test Index

The following are the indexes: flexion power (N·m), extension power (N·m), left flexion power (N·m), right flexion power (N·m), left rotation power (N·m), right Rotational power (N·m), and ratio of flexion power to extension power (flexion/extension (F/E)).

FMS is a comprehensive examination of the flexibility and stability of the human body and discovers the asymmetry and movement compensation of the human body. It can be used as a basis for formulating a functional training plan, helping to find wrong movement patterns, thereby improving sports performance. The injury played a preventive role. Observe and record the physical problems of the athletes during the test through the FMS test, analyze the test results, understand the physical condition of the athletes, and provide a basic basis for the formulation of the training plan.

#### 3.3.4. Test Methods

The specific method of functional sports inspection (FMS) testing and evaluation is to use the FMS standard test product group, which tests 7 types including squats, squats, straight supports, movable lifts, shoulder flexibility, push-ups, and rotational stability. The action will be repeated 3 times to collect the action from the front and side of the subject using the camera. Testers with the same training are rated according to the scoring standard, and the score is from 0 to 3, as shown in Table 1:

## 4. Skier Tracking Experiment and Result Analysis

### 4.1. Filtering Experimental Data Analysis

First, perform filtering experiments on the speed of skiers. The experimental data is based on randomly extracting from the database the original GPS measured speeds of skiers who glide a complete lap in the ski resort. Kalman filtering, mean filtering, and medium filtering with time series models are used, respectively. The Kalman filter selects a weighted average of the best weighting factors. Mean filtering is a typical linear filtering algorithm. The principle is to take the eight pixel points around that pixel point to take the average operation and then replace that pixel point, which is the convolution operation. Median filtering selects a fixed size sliding window and then selects the median within the sliding window as the filtering result. Or pick the median average, similar to a game where the highest and lowest scores are removed and the rest of the scores are averaged. Median filtering has a good filtering effect on impulse noise and can effectively overcome the fluctuation noise caused by accidental factors. The value filter is used to filter the speed of the skier, the ski speed filter, and the filtered results are shown in Figures 6–7.

It can be seen from Figures 6 and 7 that the overall effect of Kalman filter introduced into the time series model is not much different from the median filter and the mean filter. Both of them filter out the two obvious error deviations, but the median filter and the mean filter have a smoother effect on small disturbances, which may be distorted. The Kalman filter introduced into the time series model retains the small disturbances, which is more in line with the actual situation, and the disturbances are within the acceptable deviation range. Moreover, the median filter is filtered when the contextual ski speed is known, so it is not suitable for this project system. This project system needs to estimate the current ski speed without knowing the following ski speed. The result of the athlete's ski speed estimated by the Kalman filter with the introduction of the time series model is within the acceptable range. In the interpolation experiment of athletes' speed, the results of interpolation after Kalman filtering in Figures 6 and 7 when the sliding window length is *k* = 6 are shown in Figure 8.

After filtering and interpolating the speed of the skier, the experiment of tracking the target athlete by the dome camera needs to be carried out through PID control. The rotation speed of the dome camera deployed in the ski resort can be divided into 8 gears, of which the 1st gear is the slowest and the 8th gear is the fastest. The dome camera is driven to a suitable rotation speed according to the angle of the athlete's movement per second. Adjust the angle of the dome camera; the specific parameters are shown in Table 2.

As can be seen from Table 2, the transverse pendulum rate is 2.7 and the elevation speed is 36°/s is the maximum descent speed, reaching 4.6 m/s. When the transverse pendulum rate and elevation speed decrease, the descent speed also decreases accordingly.

### 4.2. Correlation Analysis

In order to evaluate the reliability and stability of the data used to construct the library, the FPKM value was used to analyze the correlation between the results of the two sequencing library constructions. The closer the correlation value is to 1, the better the reliability and stability, and the higher the repeatability. As shown in Figure 9, the correlation coefficient of the FPKM values of the two transcriptome libraries before and after training is 0.89, indicating that the results of the two sets of databases are relatively reliable. The calculation method of FPKM (Fragments per Kilobase Million) is the same as that of RPKM (Reads per Kilobase Million). The difference is that FPKM is used for paired-end sequencing. The 4 reads on 2 fragments are compared and calculated twice. RPKM uses coming to the single-segment sequencing library, the data (reads) are calculated, as shown in Figure 9.

As an important gene, *β*-actin gene can be quantitatively analyzed by real-time fluorescence quantitative PCR to quantitatively analyze the performance of different genes before and after high-intensity exercise, so that the increase curve of *β*-actin gene can be seen. As the number of cycle increases, there are exponential growth periods, linear growth periods, and stable periods. The melting curve results show that the temperature of each repeated melting point is the same, and the amplified products are relatively special, and there are no primer combination and other nonspecial amplified products. The temperature at which the real-time PCR product of housekeeping gene dissolves is 75°C. In the experiment, fluorescence quantitative PCR was performed on the cDNA of each Mongolian horse. The results show that although the individuals are different, the CT values of the genes are similar, all around 25, and the expression is relatively constant, as shown in Figures 10 and 11.

Among them, the following isogenes are enriched in the biological process pathway: TTN gene and PDK4 gene; TTN is the gene that encodes the myosin of the muscle node, and PDK4 plays an important function in skeletal muscle glucose metabolism. The following isogenes are enriched in the molecular function pathway: TRIM63 gene and MYL3 gene; the following is enriched in the cellular pathway isogenic genes: ACTN gene and VEGFA gene. Presumably, it is caused by changes in the body's circulatory system, binding transcription factor activity, enzyme binding, and other metabolic mechanisms due to short-term high-load exercise.

### 4.3. Experimental Results

The reason for using Hu moments as a good representation of image features is that Hu moments are geometrically invariant with respect to rotation and translation.

It is geometrically invariant in terms of rotation and translation. In order to illustrate the invariance of Hu moments in these three aspects, this paper selects the trajectory samples in the ski trajectory sample database and calculates the trajectory images after being enlarged to 4 times the original size, 75° rotation, and translation. The value of the torque-changing parameter and the calculation result are shown in Table 3.

It can be seen from Table 3 that for the 8Hu moment parameters of the image, when the image size is expanded to 4 times the original size, the two moment invariant parameters Hu3 and Hu5 change slightly. When switching or rotating at 75°, the 8Hu moment constant parameters will basically not change. This shows that within a specific allowable error range, the Hu moment of the trajectory image has good geometric invariance. In this experiment, in order to characterize the image characteristics of the trajectory, the Hu moment invariant parameter was selected. Another reason is that in a skiing competition, compared with previous movements, the position and swing of the athlete's arm each time the athlete performs an action. The rod angle cannot be completely consistent. The geometric invariance of the Hu moment parameter makes up for this shortcoming. The calculation results are shown in Table 4.

Therefore, the eight constant Hu torque parameters are derived from the trajectory samples in the sample database, as shown in Table 4, as the initial trajectory feature data recognized by the K-L transformation. Two conclusions can be drawn from Table 4. First, there are big differences between different variants of each track, so these 8-digit numbers can be used as effective feature parameters. Secondly, the Hu1~Hu7 parameters of different motion paths are quite different. Taking these eight irreversible characteristics as the 8-dimensional range of the trajectory characteristics, for the samples with the number of samples of 175, an initial data matrix of characteristics 8 to 172 is formed. The K-L transformation is carried out directly on the track samples, without the need to extract the Hu torque characteristics. The size of the original feature data matrix is 78596-125. From the scale of these two data tables, it is obvious that the amount of calculation for orbit identification is very large. Using this conversion method based on orbit characteristics greatly reduces the amount of calculation.

## 5. Conclusions

The special physical structure includes form and physiological function, which is composed of strength, endurance, and coordination training. On-land training is mainly based on multiwheel skateboarding around obstacles, while on snow is mainly based on front edge and back edge conversion and obstacle practice. Although snowboarding has been in operation for about 10 years, because the project has the characteristics of high risk, high technical level, and high requirements for competition and training venues, the degree of promotion is not high, and the number of athletes is limited. The scale of development is small, there are few ready-made theories and methods in biological monitoring and physical training, and the degree of confidentiality of research materials is high, and it is difficult to obtain data. It is recommended to highlight the characteristics of one's own items in special physical training and design more reasonable special physical training content. Skeletal muscle is an important tissue that constitutes the human body. Understanding the role of skeletal muscle in exercise can help solve the musculoskeletal system problems that may exist in different groups of people. Since the 1990s, researchers have tried to obtain muscle structural parameters such as muscle cross-sectional area, muscle thickness, pinnate angle, and muscle fiber length from ultrasound images to reflect changes in a muscle state. In addition to physiological structure, quantitative estimates of local motion can help provide more information about changes in muscle tissue during muscle contraction. This thesis mainly studies the computer-aided ultrasonic quantitative analysis of the skeletal muscle of snowboarders after exercise based on artificial intelligence and complex networks. For the motion estimation of muscle tissue, we use variational optical flow calculation to obtain the corresponding sports field. Since the split Bregman method has been widely used in image restoration, image compression, image segmentation, and other fields, we extend it to solve the problem of variational optical flow calculation. At the same time, this article only conducts preliminary tests on the gastrocnemius and quadriceps muscles, and other methods of studying skeletal muscles are needed to supplement and expand, in order to have a more complete and comprehensive understanding of skeletal muscle functions and better application in practice. Ski parallel giant slalom in China is not much research content, so the relevant theoretical technology is not mature, so the research in this paper provides part of the theoretical basis for the training of ski parallel giant slalom athletes and creates good opportunities for promotion and development in China.

## Figures and Tables

**Figure 1:** Data flow diagram-top level diagram.

**Figure 2:** Data flow diagram-0 layer diagram.

**Figure 3:** Probability distribution of the reliable class of adjacent point elements *i* and *r*.

**Figure 4:** Probability distribution of adjacent points *i* and *r* are multiple matching classes.

**Figure 5:** Ultrasound image and vector image overlay image.

**Figure 6:** The Kalman filter effect of introducing the time series model ARIMA (5,1,5).

**Figure 7:** Median filtering effect with a smoothing window size of 10.

**Figure 8:** Speed interpolation of part of the speed interval after Kalman speed filtering.

**Figure 9:** Correlation analysis of three libraries.

**Figure 10:** Amplification curve and dissolution curve of *β*-actin gene.

**Figure 11:** QRT-PCR results of upregulated and downregulated genes.

**Table 1:** FMS test score description table.

Score	Score description
3 points	Able to complete functional test actions
2 points	Able to complete functional test actions that reduce difficulty
1 points	Cannot complete the function test action
0 points	Pain in the body when completing the investigation

**Table 2:** Rotational angular velocity of the three parameters of the dome camera (unit: °/s).

Turn gear	Yaw rate	Elevation velocity	Depression velocity
1	0.5	2	0.4
2	0.6	5	0.6
3	1.2	16	2.3
4	0.9	75	2.6
5	1.8	24	3.8
6	2.7	36	4.6
7	0.9	29	3.7
8	0.7	28	2.4

**Table 3:** Hu moments of ski trajectory images under three geometric transformations.

Invariant moment parameters	The original image	4 times the size	Panning	75° rotation
Hu1	3.2561	4.5821	5.2535	4.2589
Hu2	2.5689	3.6985	6.2489	5.2655
Hu3	5.2365	5.5689	2.2587	4.2365
Hu4	5.2897	6.2583	1.6985	3.5896
Hu5	4.5823	4.5268	2.5478	2.5896
Hu6	3.5986	3.5698	3.5698	4.2563
Hu7	5.2569	2.7541	2.4789	6.5893
Hu8	4.2581	5.2369	3.2569	2.5897

**Table 4:** Values of Hu1~Hu7.

Track number	Hu1	Hu2	Hu3	Hu4	Hu5	Hu6	Hu7	Hu8
Gear trajectory 1	4.3038	5.2596	4.2587	3.2569	5.2896	4.5287	3.2569	2.9856
Gear trajectory 2	5.2698	4.5296	3.5295	4.2589	3.2569	2.8569	1.5409	1.7589
Gear trajectory 3	5.2862	7.6759	5.2365	5.2368	4.2589	3.2589	3.2569	4.2587
Gear trajectory 1	2.2135	3.2541	2.5842	3.5289	5.2658	4.8569	3.2589	3.2596
Gear trajectory 2	2.4587	3.2569	6.2589	4.5289	3.2589	6.2564	2.5879	4.5269
Gear trajectory 3	3.5298	4.2589	3.2587	2.4587	1.8569	5.2364	3.2654	5.3636

## Data Availability

The data that support the findings of this study are available from the corresponding author upon reasonable request.
